The article "A Hybrid Approach Based on Deep CNN and Machine Learning Classifiers for the Tumor Segmentation and Classification in Brain MRI" was retracted in 2023. Reasons: signs of a paper mill; compromised peer review; unreliable results or conclusions.

# A Hybrid Approach Based on Deep CNN and Machine Learning Classifiers for the Tumor Segmentation and Classification in Brain MRI

**DOI:** 10.1155/2022/6446680

**Published:** 2022-08-05

**Authors:** Ejaz Ul Haq, Huang Jianjun, Xu Huarong, Kang Li, Lifen Weng

**Affiliations:** ^1^Guangdong Key Laboratory of Intelligent Information Processing, School of Electronics and Information Engineering, Shenzhen University, China; ^2^School of Computer and Information Engineering, Xiamen University of Technology, China

## Abstract

Conventional medical imaging and machine learning techniques are not perfect enough to correctly segment the brain tumor in MRI as the proper identification and segmentation of tumor borders are one of the most important criteria of tumor extraction. The existing approaches are time-consuming, incursive, and susceptible to human mistake. These drawbacks highlight the importance of developing a completely automated deep learning-based approach for segmentation and classification of brain tumors. The expedient and prompt segmentation and classification of a brain tumor are critical for accurate clinical diagnosis and adequately treatment. As a result, deep learning-based brain tumor segmentation and classification algorithms are extensively employed. In the deep learning-based brain tumor segmentation and classification technique, the CNN model has an excellent brain segmentation and classification effect. In this work, an integrated and hybrid approach based on deep convolutional neural network and machine learning classifiers is proposed for the accurate segmentation and classification of brain MRI tumor. A CNN is proposed in the first stage to learn the feature map from image space of brain MRI into the tumor marker region. In the second step, a faster region-based CNN is developed for the localization of tumor region followed by region proposal network (RPN). In the last step, a deep convolutional neural network and machine learning classifiers are incorporated in series in order to further refine the segmentation and classification process to obtain more accurate results and findings. The proposed model's performance is assessed based on evaluation metrics extensively used in medical image processing. The experimental results validate that the proposed deep CNN and SVM-RBF classifier achieved an accuracy of 98.3% and a dice similarity coefficient (DSC) of 97.8% on the task of classifying brain tumors as gliomas, meningioma, or pituitary using brain dataset-1, while on Figshare dataset, it achieved an accuracy of 98.0% and a DSC of 97.1% on classifying brain tumors as gliomas, meningioma, or pituitary. The segmentation and classification results demonstrate that the proposed model outperforms state-of-the-art techniques by a significant margin.

The article "A Hybrid Approach Based on Deep CNN and Machine Learning Classifiers for the Tumor Segmentation and Classification in Brain MRI" was retracted in 2023. Reasons: signs of a paper mill; compromised peer review; unreliable results or conclusions.

## 1. Introduction

Brain tumors are lumps that arise as a result of aberrant brain cell proliferation and the loss of the brain's regulatory systems. Tumors in the head cranium can grow and strain on the brain, affecting physical health. Early tumor segmentation is an essential research topic in medical imaging's field since it helps doctors choose the best treatment strategy for a patient's health. Over the last several decades, medical researchers have found more than 120 different kinds of brain tumors. There are two types of brain tumors: primary brain tumors that form in the brain and secondary brain tumors that can be found in the brain but arise elsewhere in the body [1]. Brain tumors become more common as people get older [1]. Gliomas, meningioma, and pituitary brain tumors are the main focus of this research. The World Health Organization divides gliomas into I-IV categories based on their location, type, and tumor size. Low-grade gliomas are classified as classes I and II, whereas high-grade gliomas are classified as classes III and IV [2].

In most cases, noninvasive medical imaging methods such as computer tomography (CT) and MRI are preferred over invasive procedures for brain tumor segmentation of gliomas, meningioma, and pituitary tumors, allowing clinicians to safely remove tumors within the maximum range [3]. As a result, tumor segmentation is considered the initial step in the analysis of MRI of infected people. Manual segmentation of tumor areas takes a long time and a lot of effort because tumors have varying degrees of degradation and include many tissue regions. Furthermore, the overall employment of diagnostic imaging system and MRI technicians is increasing at a higher rate than the average [4]. All of these findings support the notion that medical image-based diagnostics is preferred in today's healthcare sector.

Furthermore, manual segmentation is frequently dependent on the intensity of the image as seen by the human eye, which can be easily influenced by the image quality as well as observer personal observations. It is susceptible to incorrect segmentation and redundant area segmentation. However, the following are the issues that have been identified in the investigation of automated glioma segmentation methods: (1) the difference in pixel intensity between the tumor region and surrounding normal tissues is commonly used to identify brain tumor in images. The intensity differential between neighboring tumor tissues will be flattened due to the existence of a gray-scale field, which will result in blurry tumor borders. (2) It is challenging for image segmentation methods to clearly diagnose the brain tumor as the size, structure, and location of tumor vary [5]. As a result, in clinical practice, a fully automated tumor segmentation approach with high accuracy is required.

The article "A Hybrid Approach Based on Deep CNN and Machine Learning Classifiers for the Tumor Segmentation and Classification in Brain MRI" was retracted in 2023. Reasons: signs of a paper mill; compromised peer review; unreliable results or conclusions.

Over the last two decades, medical image segmentation and classification have improved drastically with the advancement in machine learning and computer vision techniques. In recent years, machine learning-based computer-aided diagnostic technology has grown in popularity in medical imaging [6]. Machine learning technique can solve classification, regression, and segmentation problems in medical images because it can train model parameters using distinct features of medical images and then use the learned model to predict the extracted features. Methods for segmenting brain tumors may be generally grouped into three types: conventional imaging algorithms, machine learning-based techniques, and methods utilizing DL networks.

Deep learning has been applied in medical imaging to identify cells of various sizes and shapes, identify organs and body components, and detect local anatomical features [2]. Deep learning can have a big influence with encouraging outcomes on medical image segmentation and classification. It makes noninvasive imaging-based diagnostics more automated [7]. This study focuses on the glioma, meningioma, and pituitary segmentation and classification technique, which uses a deep learning algorithm to automatically and correctly separate the tumor region from a brain MRI and then classify it. In this work, we have described an automated method for segmenting and classifying the brain tumor including glioma, meningioma, and pituitary in MRI images. The following are the key research contributions covered in this paper:

1. A hybrid and integrated classifier based on deep CNN and machine learning classifiers, i.e., random forest (RF), support vector machine-RBF (SVM-RBF), and extreme learning machine (ELM), is proposed for the accurate segmentation and classification of brain tumor into glioma, meningioma, and pituitary tumor. Image registration approach is adopted in the preprocessing of brain MRI scans. The brain MRI images were either linearly or nonlinearly register, merely cropped or padded to the required size. In comparison to no image registration, both linear and nonlinear registration improves the accuracy of the classifier by about 4-5 percent. The performance of the classifier is improved by image registration, although the choice of linear or nonlinear image registration has minimal effect on segmentation and classification accuracy. In the first stage, a CNN is developed to learn the feature map from brain MRI image space into the tumor marker area. The proposed CNN is trained using 3 separate preprocessed brain MRI scans. In the second step, a region-based CNN is proposed for tumor localization, preceded by a region proposal network (RPN). One of the most important problems in medical image processing is the lack of labeled data. As a result, the focus of our research on employing R-CNN-based tumor localization in scenarios when annotated data is limited. We extended the segmentation and classification procedure to build the structure of the next deep CNN and machine learning classifiers in series in order to improve the accuracy of segmentation and classification output
2. As part of this research, we were able to provide an end-to-end, systematic method for brain tumor segmentation and classification utilizing brain MRI. The system composed of three parts: brain tumor segmentation with a basic CNN algorithm, tumor localization with a faster R-CNN-based network, and exact tumor segmentation and classification using a deep CNN and machine learning classifier framework. The final outcome of all three algorithms was the exact tumor boundary, which was categorized into glioma, meningioma, and pituitary tumor types
3. The experimental results validate that the proposed deep CNN and SVM-RBF classifier achieved an accuracy of 98.3% and a dice similarity coefficient (DSC) of 97.8% on the task of classifying brain tumors as gliomas, meningioma, or pituitary using brain dataset-1, while on Figshare dataset, it achieved an accuracy of 98.0% and a DSC of 97.1% on classifying brain tumors as gliomas, meningioma, or pituitary

The rest of the paper is organized in the following way: Section 2 briefly summarizes the related research.

The article "A Hybrid Approach Based on Deep CNN and Machine Learning Classifiers for the Tumor Segmentation and Classification in Brain MRI" was retracted in 2023. Reasons: signs of a paper mill; compromised peer review; unreliable results or conclusions.

The proposed method is described in Section 3. The performance analysis using objective matrices is presented in Section 4.  Section 5 shows comparison of our proposed method to prior studies in the literature.  Section 6 discusses the conclusion.

## 2. Related Research

Artificial intelligence are largely utilized in image processing techniques for segmenting, identifying, and classifying MRI images, as well as for classifying and detecting brain cancers. There have been several studies on the classification and segmentation of brain MRI images. These technologies use techniques such as conventional image processing and a machine learning approaches based on neural networks to diagnose brain cancers. The authors in [8] utilized the multilayer perceptron (MLP) to categorize brain tumors as normal or abnormal with an accuracy of 85% and support vector machine (SVM) with an accuracy of 74% to classify brain tumor. The authors of [9] presented a technique for identifying brain lesions in which the tumor is first segmented from an MRI image and then extracted using stochastic gradient descent by a pretrained convolutional neural network. Shahriar et al. [10] propose an approach that uses Matrix Laboratory (MATLAB) to equip threshold-based Otsu's segmentation, which identifies the tumor and segments the tumor site with an accuracy of 95%. Selvaraj et al. [11] developed a binary classifier utilizing first-order and second-order statistics and a least square support vector machine (SVM) to identify normal and malignant MRI brain scans. The authors in [12] propose an automated system based on a feed-forward neural network with back-propagation, used to identify brain tumors. This has a 99 percent accuracy rate. Sajjad et al. [13] utilized a data augmentation approach on brain MRI scans and then adjusting it with a pretrained VGG-19 CNN model to classify multigrade tumors. Carlo et al. [14] used multinomial logistic regression and k-nearest neighbor techniques to develop a method for detecting pituitary adenoma tumors. The approach achieved an accuracy of 83% on multinomial logistic regression and 92% on a k-nearest neighbor with an AUC curve of 98.4%. Gurbină et al. [15] used a hybrid approach based on CWT, DWT, and SVMs to identify brain tumors, segment them, and categorize them based on malignancy. In this method, several wavelet levels were employed, and CWT achieved high accuracy. Dvorak et al. [16] developed a multimodal MRI-based automated tumor detection approach that includes skull extraction from a T2-weighted image, image cutting, anomaly probabilistic map computation, and feature extraction to identify a brain tumor. Initially, this method produces an average accuracy of 90%. The shape deformation feature has the potential to increase segmentation quality. Khawaldeh et al. [17] developed a framework based on the Alex-Net CNN model for classifying brain MRI images into healthy and unhealthy, as well as a grading system for categorizing unhealthy brain MRI images into low and high grades. The proposed Alex-Net CNN model achieved accuracy of 91%. Ezhilarasi and Varalakshmi [18] considered using a bounding box to detect the brain tumor area and determine the type of tumor. Using the proposed method, the tumor is categorized as malignant, benign, glial, or astrocytoma. A faster region-based CNN was used to train brain MRI images from scratch, and the obtained results were impressive. Several studies have recently presented numerous approaches for detecting and segmenting the tumor area using brain MRI images [19, 20]. Once tumor region in MRI scans has been segmented, then it can be classified into distinct grade tumors. Binary classifiers have been used in earlier research studies to distinguish between benign and malignant classes [21–23]. Ullah et al. [21] presented a hybrid approach utilizing histogram equalization, DWT, and feed-forward ANN for classifying brain MR images into normal and abnormal. Kharrat et al. [22] presented a machine learning approach based on genetic algorithm and support vector machine for classifying brain tumors into normal and abnormal group.

The article "A Hybrid Approach Based on Deep CNN and Machine Learning Classifiers for the Tumor Segmentation and Classification in Brain MRI" was retracted in 2023. Reasons: signs of a paper mill; compromised peer review; unreliable results or conclusions.

Furthermore, Papageorgiou et al. [23] used fuzzy cognitive maps to classify high-grade and low-grade gliomas, achieving 93.22% and 90.26% accuracy for high-grade and low-grade brain tumors, respectively. Das et al. [24] used an image processing approach to train a CNN model to identify different brain tumor types, achieving 94.39 percent accuracy and 93.33 percent precision. Deep learning algorithms have been widely utilized for brain MRI classification during the last decade [25, 26]. Because the feature extraction and classification stages are incorporated in self-learning, the deep learning approach does not require manually derived features. The deep learning approach necessitates a dataset, which may require some preprocessing, before significant characteristics are selected in a self-learning way [27]. Mzoughi et al. [28] used a 3-dimensional brain MRI image for the classification of low-grade glioma and high-grade glioma based on deep multiscale 3D CNN model that achieved classification accuracy of 96.49%. The authors in [29] presented a CNN-based approach with data augmentation for classifying brain tumors as malignant or nonmalignant using 253 brain MRI scans. They used edge detection to find the region of interest in an MRI image before extracting the data with a basic CNN model. They were able to attained 89% classification accuracy. A combined feature-image-based classifier (CFIC) is presented in [30] for the classification of brain tumor images. The designs are based on deep convolutional neural networks (DCNN) and deep neural networks (DNN) for image classifications. In [31], two models, ResNet (2 + 1)D and ResNet Mixed Convolution, are used to distinguish between different types of brain cancers. In both of these models, the performance was better than ResNet18, a 3D convolutional network. Additionally, if models are pretrained on a different dataset before being trained to classify tumors, performance is enhanced. In [32], min-max normalization and a dense efficient net-based CNN were employed to classify 3260 T1-weighted contrast-enhanced brain magnetic resonance images into four groups (gliomas, meningiomas, pituitary, and no tumor). The authors in [33] compared various models of automated brain tumor cell prediction, including CNN-trained VGG-16, ResNet-50, and Inception-v3. The dataset contains 233 images of MRI brain tumors, which were used to train the pretrained models. In conclusion, the obtained accuracies utilizing deep learning approaches for brain MRI classification are significantly higher than conventional ML techniques, as shown in the previous research findings. Deep learning algorithms need a significant amount of training data in order to outperform traditional ML approaches. Techniques based on deep learning have definitely become one of the primary streams of expert and intelligent systems and medical image analysis, as evidenced by recently published research.

The article "A Hybrid Approach Based on Deep CNN and Machine Learning Classifiers for the Tumor Segmentation and Classification in Brain MRI" was retracted in 2023. Reasons: signs of a paper mill; compromised peer review; unreliable results or conclusions.

## 3. Proposed Model

The overall architecture of our proposed framework is presented in this section. The contents of four important components are then described in the subsections.  Figure 1 depicts the architecture of our proposed framework for brain tumor segmentation and classification. Before being fed into the model, incoming MRI scans are first preprocessed using image registration phenomena. Preprocessed brain MRI scans are fed into CNN, which uses them to learn a feature map from brain MRI image space to the tumor marker region. In next step, a region-based CNN is proposed for tumor localization, followed by an RPN. To enhance the accuracy of the brain tumor segmentation and classification results, we expanded the segmentation process to create the structure of the next deep CNN and machine learning classifiers in series.

### 3.1. Preprocessing Using Image Registration

Preprocessing is used to enhance image data by removing undesirable distortions and improving specific visual features that are important for subsequent processing. Image registration is a type of image processing that combines several scenes into a single image. When overlaying images, it helps to overcome problems such as image rotation, size, and skew. The process of converting multiple images into the same coordinate system with matching imaging information is known as image registration. It is been used in a variety of clinical settings and medical research. The images to be recorded may be obtained for the same subject using multiple modalities, in the same modality but from separate subjects, or in the same modality but from the same subject at a different time, depending on the medical reasons. For time series analysis or longitudinal investigations, registration may also be done on images recorded over time.

In this work, the brain MRI scans were only registered to linear or nonlinear template, cropped or padded to needed size. It has been showed that image registration increases the accuracy of classifier by about 4-5 percent compare to no image registration. The affine transformation was used to directly align data from each sample to the MNI template, resulting in linear registration. Transformations (*T*_(*y* − *z*)_) were acquired using AIR, which was deployed to each patient's brain mask for dice coefficient measurement.  Figure 2 shows linear registration. Because the MR images in our dataset have varying widths, heights, and sizes, it is essential that they have to be resized to the same width and height to achieve the best results. We reduce the MR images 224 × 224 pixels in this study since the input image dimensions of CNN models are 224 × 224 pixels.

The article "A Hybrid Approach Based on Deep CNN and Machine Learning Classifiers for the Tumor Segmentation and Classification in Brain MRI" was retracted in 2023. Reasons: signs of a paper mill; compromised peer review; unreliable results or conclusions.

### 3.2. Feature Extraction Using CNN Models

CNNs are a type of deep neural network that processes inputs for relevant information utilizing convolutional layers. Convolutional filters are applied to the input by CNN's convolutional layers, which compute the output of neurons linked to particular areas in the input. It aids in the extraction of image spatial and temporal information. In the convolutional layers of CNN, a weight-sharing approach is utilized to minimize the overall number of parameters.

In this work, a CNN-based model as a feature extractor is employed since it can extract key features without the need for human interference. The proposed CNN structure is shown in Figure 3, and it comprises of three convolutional layers, each followed by a max-pooling layer and lastly a fully connected layer. The output is either tumor or no tumor. A convolutional kernel of size 7 × 7 is multiplied on each input image. For the first, second, and third convolutional layers, same convolutional kernel of size 3 × 3 is used, as well as filter sizes of 32, 64, and 128 for the first, second, and third layers, respectively. A kernel size of 2 × 2 is used in each pooling layer. The final output segmentation results are generated by the fully connected layer at the network's end.

### 3.3. Faster R-CNN with Region Proposal Network for Tumor Localization

The R-CNN is a tracking and localization method based on neural network architecture. It uses a recognition-based segmentation methodology. It first extracts free-form region of interest (ROI) from the input image, then executes region-based segmentation on those ROI. Region based-CNN and RPN [34] are the two major subnetworks that make up the faster R-CNN. RPN reduces the number of search regions through generating anchors in an image, and it works as a classifier, training CNNs how to categorize selected ROIs or region proposals into object classes. R-CNN begins by segmenting an input image into several subimages called regions, each with a distinct dimension. Each region is then treated as a separate image, which is subsequently categorized into a series of predetermined object categories. Finally, by integrating subimages with comparable regions, region proposals with projected object labels are created. R-CNN selects these ROIs using selective search methods, which results in a high computation complexity and slow processing time because it creates over 2000 areas for each input image. Because the cost of creating region proposals in RPN is significantly lower than in the selective search technique, the RPN-based bounding box detection method was added to faster R-CNN. The primary difference between R-CNN and faster R-CNN is that the former uses pixel-level region proposals while the latter uses feature map-level region proposals. RPN creates 9 anchors from the input image and predicts whether an anchor will be in the background or front. These anchors are given positive or negative labels depending on two major indicators. Anchors having a greater intersection-over-union (IOU) are found to belong to the ground truth box. As a consequence, the anchor target obtains a positive label if the IOU overlap between an anchor and ground truth is more than 0.7, but the area receives a negative label if it is less than 0.3. Learning is not done with anchors with IOU values between 0.3 and 0.7. In the RPN network's training phase, the loss function in (1), which is defined using the values provided to the anchors, is used:

(1) $$\begin{array}{c} L\left(\left\{p_{j}\right\},\left\{v_{j}\right\}\right)=\frac{1}{M}\underset{j}{\sum }S_{L}\left(p_{j},p_{j}^{\prime }\right)+\delta \frac{1}{P}\underset{j}{\sum }p_{j}^{\prime }R_{L}\left(v_{j},v_{j}^{\prime }\right), \end{array}$$

where *p*_*j*_ represent the anchor's predicted probability, *j* shows the anchors index, *v*_*j*_ is a vector which represent the four coordinates of identified bounding box, *M* represents the total size of minibatch, *S*_*L*_ is the segmentation loss, *P* shows the location of anchor, and *R*_*L*_ represent regression loss. *p*_*j*_′ represents the positive anchors, and its value is assigned 1 when object lies inside anchor. The value 1 is assigned based on algorithm. *v*_*j*_′ stands for the ground truth box, which is related to a positive anchor.  Figure 4 depicts the region proposal network.

The article "A Hybrid Approach Based on Deep CNN and Machine Learning Classifiers for the Tumor Segmentation and Classification in Brain MRI" was retracted in 2023. Reasons: signs of a paper mill; compromised peer review; unreliable results or conclusions.

### 3.4. Deep CNN and Machine Learning Classifiers

The segmentation and classification process is improved, and an iterative technique is used to connect the CNN and the interconnected machine learning classifiers such as random forest, SVM-RBF, and extreme learning machine to increase the accuracy of the results. After extracting the bounding box using the proposed faster R-CNN based model, a deep CNN and machine learning classifiers are used to produce a precise tumor boundary. The localized tumor is classified into three groups after segmentation: glioma, meningioma, and pituitary.

Each convolutional layer is followed by a max-pooling layer and eventually a fully connected layer in the proposed CNN. A convolutional kernel of size 7 × 7 is multiplied on each input image. For the first, second, third, and fourth convolutional layers, same convolutional kernel of size 3 × 3 is used, as well as filter sizes of 32, 64, 128, and 256 for the first, second, third, and fourth layers, respectively. A kernel size of 2 × 2 is used in each pooling layer. The segmented output of fully connected layer is further given to machine learning classifier for the classification of segmented tumor into glioma, meningioma, and pituitary. The final step is repeated again to refine the segmentation and classification results.  Figure 5 shows the framework of deep CNN and machine learning classifiers.

#### 3.4.1. Convolutional Layer

For the segmentation and classification process, convolutional layers create a feature map for each point of the input MRI image. Neurons are the most basic and important component of the convolutional layer that creates the feature map. Although all neurons in the feature map must have identical weights, different feature maps result in varied weights in the same convolutional layer, allowing for the extraction of several features at each and every location. Each convolutional layer uses ReLu as an activation function.

#### 3.4.2. Pooling Layer

The major objective and goal of the pooling layer is downsampling, i.e., reducing the resolution and size of the feature map produced from the convolutional layer. Average pooling and maximum pooling are the two most prevalent pooling techniques. The originality of the input image is reduced by the average pooling layer, but the originality of the source image is preserved by the max-pooling layer. The highest value of the feature map is also preserved by the max-pooling layer, which is why it is the major subject of the research. Kernel size of 2 × 2 and stride of 2 is deployed in the max-pooling layer.

#### 3.4.3. Fully Connected (FC) Layer

Following the convolutional layer and max-pooling, the FC layer includes final classification results with distinct classes. In the fully connected layer, a dropout probability of 0.5 is utilized to minimize overfitting problems, and softmax was used as an activation function. The CNN network's layers receive training and testing samples from the previous layer and pass them along to the next layer. Finally, the fully connected layer takes input from the previous max-pooling layer and classifies the feature map into subclasses.

The article "A Hybrid Approach Based on Deep CNN and Machine Learning Classifiers for the Tumor Segmentation and Classification in Brain MRI" was retracted in 2023. Reasons: signs of a paper mill; compromised peer review; unreliable results or conclusions.

The loss function is used to compute the loss, which is the neural network's prediction error. The loss is utilized to calculate the gradients and update the weights of the neural network in the training step. The cross-entropy loss function, which is the most widely used loss function in convolutional neural network, is utilized in the FC classifier's training phase. It estimates the difference between the ground-truth label and the soft target calculated by the softmax function and can be expressed as

(2) $$\begin{array}{c} L\left(v,w\right)=\overset{N}{\underset{j=0}{\sum }}-v_{j}\log\left(\frac{w_{i}}{\sum_{k}\exp\left(w_{i}\right)}\right), \end{array}$$

where *N* represents the total number of classes, *v* is vector which shows the ground truth label, and *w*_*i*_ represent the output of last layer.

#### 3.4.4. Random Forest

Breiman [35] introduced RF, an ensemble learning technique that uses the bagging approach to categorize new data instances to a class target of brain tumor (normal, glioma tumor, meningioma tumor, and pituitary tumor). When building decision trees, RF chooses *n* random characteristics or features to determine the best splitting position using the Gini index as a cost function. This random selection of characteristics or features helps minimize ensemble error rates by reducing correlation among trees. New attributes and features are given as input to random forest classification tree in order to forecast the class target. Total number of predictions is calculated for each class, and class having most predictions is selected as label for new entity. When exploring the optimum split, the set of features to examine is limited to the square root of the entire number of characteristics. A total number of trees are set from 1 to 150 and choose tree having best accuracy.

#### 3.4.5. Support Vector Machine-RBF

Cortes and Vapnik [36] proposed SVM as one of the most powerful classification methods. SVM classifier works on basis of hyperplane that separate two groups by the maximum possible margin. SVM employs the kernel function to transform the original data space into a higher-dimensional space. In this study, kernel RBF, the most frequently used kernel function, is employed in SVM. SVM also contains two important hyperparameters: C and gamma. C is the soft margin cost function's hyperparameter that regulates the impact of each support vector. Gamma is a hyperparameter that controls the amount of curvature in a decision boundary. We chose the combination of gamma and C values with the best accuracy by setting them to [0.00001, 0.0001, 0.001, 0.01] and [0.1, 1, 10, 100, 1000, 10000], respectively. The function for separating data can be expressed as

(3) $$\begin{array}{c} F\left(v_{j}\right)=\overset{M}{\underset{i=1}{\sum }}\sigma_{i}z_{i}K\left(v_{i},v_{j}\right)+c, \end{array}$$

where *K*(*v*_*i*_, *v*_*j*_) represents the kernel function, *v*_*j*_ shows deep features of brain tumor MRI in the form of vector data, *z*_*i*_ is the target class, and *σ*_*i*_ represents Lagrange multipliers.

The article "A Hybrid Approach Based on Deep CNN and Machine Learning Classifiers for the Tumor Segmentation and Classification in Brain MRI" was retracted in 2023. Reasons: signs of a paper mill; compromised peer review; unreliable results or conclusions.

#### 3.4.6. Extreme Learning Machine

The extreme learning machine (ELM) is a fundamental learning algorithm for feed-forward neural networks with a single hidden layer (SLFNs). Huang et al. [37] first developed ELM to address the shortcomings of classic SLFN learning algorithms, such as inferior generalization efficiency, inappropriate variable adjustment, and poor training performance. ELM has demonstrated a high level of competence in regression and classification tasks, as well as a high level of adaptability. The following is a mathematical formulation for an extreme learning machine:

(4) $$\begin{array}{c} Mv=T, \end{array}$$

where *M* shows the hidden layer output matrix, the weighted vector is denoted by *v*, while the required output matrix is denoted by *T*. The fundamental goal of the extreme learning machine technique is to select the optimal strategy for *v*, which is then utilized to minimize the gap between the network's estimated and actual outputs. If the training dataset and hidden nodes are identical, *M* will be a square matrix. The input weights and hidden layers are hard to distinguish if *M* is a nonsquare matrix though.

## 4. Experiments and Results

### 4.1. Dataset Preparation

We conduct a series of experiments using three publicly accessible brain MRI datasets for the segmentation and classification of brain tumors. The first dataset was obtained from the Kaggle website [38] which contain total of 3174 brain MRI images, and we called it brain dataset-1 for simplicity. Brain dataset-1 comprises total 2674 tumor images and pituitary and 500 nontumor images. Brain dataset-1 includes 926 glioma scans, 937 meningioma, and 901 pituitary tumors among the 3174 images. The 2nd dataset utilized in this work is Figshare [39] comprising a total of 3064 T1-weighted contrast-enhanced brain MRI images which were obtained from 233 individuals. Gliomas, meningioma, and pituitary tumors were the three primary kinds of brain tumor MRI images included in this dataset. Figshare dataset includes 1426 glioma scans, 708 meningioma, and 930 pituitary tumors among the 3064 images. Each dataset is further split into a training set (75 percent of the entire dataset) and a test set (25 percent of the entire dataset). Tables 1 and 2 describe the training and testing details using the brain dataset-1 and the Figshare dataset, respectively.

The article "A Hybrid Approach Based on Deep CNN and Machine Learning Classifiers for the Tumor Segmentation and Classification in Brain MRI" was retracted in 2023. Reasons: signs of a paper mill; compromised peer review; unreliable results or conclusions.

The Adam optimizer (adaptive moment estimation), a technique for stochastic optimization, was used to train our model using 100 epochs and a learning rate of 0.00001.  Table 3 shows the hyperparameter values.

### 4.2. Performance Analysis

The proposed model's performance and efficiency were validated using evaluation measures. The four primary and fundamental metrics frequently used to evaluate the performance are true negative (tn), true positive (tp), false positive (fp), and false negative (fn). Specificity, sensitivity, PPV (positive predicted value), NPV (negative predicted value), accuracy, and dice similarity coefficient (DSC) are the classification performance evaluation metrics of the proposed model. Mean square error (MSE), peak signal-to-noise ratio (PSNR), boundary displacement error (BDE), variation of information (VOI), probabilistic random index (PRI), and global consistency error (GCE) are the segmentation performance evaluation metrics.

#### 4.2.1. Sensitivity

The capability of a model to properly identify relevant brain tumors can be expressed as follows:

(5) $$\begin{array}{c} \text{Sensitivity}=\frac{\text{tp}}{\text{tp}+\text{fn}}\times 100\%. \end{array}$$

#### 4.2.2. Specificity

The ability of a model to properly detects and classifies an actual brain tumor can be expressed as

(6) $$\begin{array}{c} \text{Specificity}=\frac{\text{tn}}{\text{tn}+\text{fp}}\times 100\%. \end{array}$$

#### 4.2.3. PPV (Positive Predicted Value)

PPV (positive predicted values) and precision are similar. It calculates true positive measures, which can be computed using the formula below.

(7) $$\begin{array}{c} \text{PPV}=\frac{\text{tp}}{\text{tp}+\text{fp}}\times 100\%. \end{array}$$

#### 4.2.4. NPV (Negative Predicted Value)

The probability of the absence of a brain tumor based on actual negative value can be computed as

(8) $$\begin{array}{c} \text{NPV}=\frac{\text{tn}}{\text{tn}+\text{fn}}\times 100\%. \end{array}$$

#### 4.2.5. Accuracy

It refers to the system's capacity to distinguish between different forms of brain tumors. The following formula was used to determine accuracy:

(9) $$\begin{array}{c} \text{Accuracy}=\frac{\text{tp}+\text{tn}}{\text{tp}+\text{tn}+\text{fn}+\text{fp}}\times 100\%. \end{array}$$

#### 4.2.6. Dice Similarity Coefficient (DSC)

It is a performance metric that can be used to assess sample overlap and can be written as

(10) $$\begin{array}{c} \text{DSC}=\frac{2\text{tp}}{2\text{tp}+\text{fp}+\text{fn}}\times 100\%. \end{array}$$

The article "A Hybrid Approach Based on Deep CNN and Machine Learning Classifiers for the Tumor Segmentation and Classification in Brain MRI" was retracted in 2023. Reasons: signs of a paper mill; compromised peer review; unreliable results or conclusions.

#### 4.2.7. Mean Square Error (MSE)

It represents the average squared difference between actual and predicted value and can be expressed using following expression:

(11) $$\begin{array}{c} \text{MSE}=\frac{1}{m}\overset{m}{\underset{j=1}{\sum }}{\left(X_{i}-\overset{\wedge }{X_{i}}\right)}^{2}, \end{array}$$

where *m* represents the total image's sample, $\hat{X_{i}}$ denotes the predicted image, and *X*_*i*_ represents the actual image.

#### 4.2.8. Peak Signal-to-Noise Ratio (PSNR)

The ratio of a signal's maximum power to the signal's maximum noise power is what it is called PSNR. PSNR is calculated using peak signal power. The PSNR is expressed in decibels. Let us assume *f* represents the original image and *g* represents the segmented and classified image.

(12) $$\begin{array}{c} \text{PSNR}=20\log_{10}\frac{P^{2}}{\sqrt{1/XY\sum_{i=0}^{X}\sum_{i=0}^{Y}{\left[f\left(i,j\right)-g\left(i,j\right)\right]}^{2}}}. \end{array}$$

*M* and *N* represent the image's size, while *P* denotes the image's pixels. A higher PSNR number implies a higher quality. PSNR is an excellent quality indicator for white noise interference.

#### 4.2.9. Boundary Displacement Error (BDE)

The average displacement error between the projected border pixels and the ground truth pixel and can be calculated as follows:

(13) $$\begin{array}{c} \partial \left(x,y\right)=\left\{\frac{x-y}{L-1}\right., \end{array}$$

where *∂*(*x*, *y*) denotes the fuzzy relation.

#### 4.2.10. Variation of Information (VOI)

It calculates the distance between the two segmentations in terms of information. The entropy and mutual information are used to define VOI:

(14) $$\begin{array}{c} \text{VOI}\left({\text{FS}}_{x},{\text{FS}}_{y}\right)=E\left({\text{FS}}_{x}\right)+E\left({\text{FS}}_{y}\right)-2M\left({\text{FS}}_{x},{\text{FS}}_{y}\right), \end{array}$$

where FS_*x*_ and FS_*y*_ denote the image fuzzy segmentation, entropy is represented by *E*(FS), *E*(FS_*x*_, FS_*y*_) denotes the combined entropy of two images, and *M*(FS_*x*_, FS_*y*_) represents the mutual information of two images.

#### 4.2.11. Probabilistic Random Index (PRI)

It is a metric for the algorithm's rate of success in making accurate predictions. The following formula can be used to calculate it:

(15) $$\begin{array}{c} \text{PRI}=\frac{\text{tp}+\text{tn}}{\text{tp}+\text{tn}+\text{fn}+\text{fp}}. \end{array}$$

*(1) Global Consistency Error (GCE)*. The GCE determines how much one segmentation may be considered a refinement of another, because they might reflect the same image segmented at various scales. GCE is calculated using the following formula:

(16) $$\begin{array}{c} \text{GCE}\left(S_{x},S_{y}\right)=\frac{1}{m}\min\left(\underset{j}{\sum }E\left(S_{x},S_{y},p_{i}\right),\underset{j}{\sum }E\left(S_{y},S_{x},p_{i}\right)\right), \end{array}$$

where *S*_*x*_ and *S*_*y*_ denote two segmentations and *p*_*i*_ represent position of pixel.

The article "A Hybrid Approach Based on Deep CNN and Machine Learning Classifiers for the Tumor Segmentation and Classification in Brain MRI" was retracted in 2023. Reasons: signs of a paper mill; compromised peer review; unreliable results or conclusions.

### 4.3. Experimental Results

The experimental findings clearly show that increasing the system structure and complexity increased the proposed model's efficiency. In terms of texture and intensity, each tumor type belonging to a particular class differs considerably from other tumor type belonging to the same class. The proposed deep CNN and machine learning classifiers can segment and categorize different types of brain tumors, regardless of their appearance or contrast. We compared the effectiveness of the developed deep CNN and ML classifiers on the brain dataset-1 and the Figshare dataset. Tables 4 and 5 demonstrate the evaluation metrics for deep CNN and machine learning classifiers on brain dataset-1 and Figshare datasets, respectively, in terms of sensitivity, specificity, PPV, NPV, accuracy, and DSC.  Table 6 shows the average overall performance of the deep CNN and machine learning classifiers on brain dataset-1 and Figshare dataset with and without image registration. It can be observed from the obtained results in Tables 4–6 that the proposed deep CNN and SVM-RBF classifier outperforms the remaining two models on the basis of different evaluation metrics.

Figure 6 shows the detected and classified results obtained based on deep CNN and SVM-RBF classifier. Figures 7 and 8 show the area under the receiver operating characteristic (AUC ROC) curves for different tumor classes in brain dataset-1 and Figshare dataset, respectively.

Figures 9 and 10 show the segmentation performance of the proposed deep CNN and machine learning classifiers on brain dataset-1 and Figshare dataset in terms of MSE, PSNR, BDE, VOI, PRI, and GCE, respectively.

Figure 11 demonstrates the graphical representation of accuracy and loss of the proposed deep CNN SVM-RBF method. Our proposed model is able to learn high-dimensional data on smaller epoch's value. As the number of epochs increases, the training and testing losses decrease, resulting in increased accuracy. It illustrates the model's increased capacity to anticipate.

## 5. Comparison of the Proposed Method with the State-of-the-Art Techniques

In this part, we compare our proposed technique to prior research that employed the same types of brain tumors but different network topologies and parameters.  Table 6 shows the results of the comparison study, which demonstrate that our proposed network achieved state-of-the-art accuracy and provided the best classification result among the techniques investigated, confirming the model's robustness and reliability. Francisco et al. [40] presented a multipath approach based on CNN for the automated segmentation of glioma, meningioma, and pituitary tumor in the brain. They tested their model against a publicly accessible MRI dataset and found it to be 97.3% accurate. Their training, on the other hand, is extremely costly. Çinar and Yıldırım [41] utilized several CNN architectures to categorize brain MRI. They tested well-known CNN models including GoogLeNet, Inception V3, DenseNet-201, AlexNet, and ResNet-50 and determined all to be effective sufficient. They achieved highest accuracy of 97.2% by modifying the last 5 layers of ResNet-50 and adding 8 new layers, as a result attained highest accuracy among other pretrained CNN models. Hemanth et al. [42] proposed a CNN-based approach for the classification of brain MRI into normal and abnormal. They utilized 220 brain MR images and attained classification accuracy of 94.5%. The authors of [43] devised a CNN network model for utilizing MRI data to classify brain tumors into distinct groups. The proposed model emphasized on complex patterns with modified activation functions. A collection of 1426 glioma images, 708 meningiomas, and 930 pituitary images were utilized. The developed model achieved 95.49% accuracy on the objective of categorizing brain tumors into three groups. Saxena et al. [44] utilized Inception V3, ResNet-50, and VGG-16 networks using transfer learning techniques to categorize brain tumor. ResNet-50 model came out on top with 95% accuracy rate. Ayadi et al. [45] proposed a robust approach for automated brain tumor classification, which is successful in extracting key characteristics from the MRI dataset by using 3 × 3 kernels in convolutional layers. The new model achieves accuracy of 94.74% in brain tumor classification with minimal preprocessing. Ghassemi et al. [46] developed a novel deep learning approach for MRI image tumor classification. They developed an unsupervised pretraining technique based on deep neural networks to address the problem of overfitting using GAN. The most robust features are extracted, and the whole structures of MR images are learned in the convolutional layer of deep neural network. The entire deep neural network is trained as classifier to identify three tumor types and attained accuracy of 93.01%. Ozyurt et al. [47] presented a brain tumor detection method that combined fuzzy C-means with superresolution and CNN with extreme learning machine methods (SR-FCM-CNN). The objective of this study was to employ the superresolution fuzzy-C-means (SR-FCM) technique to accurately segment tumors from brain MR images for tumor identification. The developed approach attained accuracy of 95.62% on 500 MR images taken from TCGA-GBM database. Sultan et al. [48] developed a deep CNN model for the categorization of brain tumors utilizing brain MRI dataset of 3064 images. The proposed model is used to categorize tumors as gliomas, meningiomas, or pituitary tumors. The deep learning model attained an accuracy of 96.13% on the task of identifying tumors as gliomas, meningiomas, or pituitary. Deep learning approaches have definitely become one of the primary streams of expert and intelligent systems and medical image analysis, as evidenced by recently published research.  Table 7 shows a comparison of the proposed methodology with the studies that have already been published. Our developed approach produced robust classification results, but more data and information about the patients, such as age, race, and health condition, are needed for testing, which might expand the applicability of the presented scheme to other therapeutic diagnostics and clinical applications.

The article "A Hybrid Approach Based on Deep CNN and Machine Learning Classifiers for the Tumor Segmentation and Classification in Brain MRI" was retracted in 2023. Reasons: signs of a paper mill; compromised peer review; unreliable results or conclusions.

## 6. Conclusion and Future Work

In this paper, a hybrid and integrated classifier based on deep convolutional neural networks and machine learning classifiers is proposed to improve segmentation and classification accuracy and achieve automatic segmentation and classification of brain tumors in MR images into glioma, meningioma, and pituitary without user intervention. The preprocessing of brain MRI images uses an image registration technique. The brain MRI images were either registered linearly or nonlinearly or simply cropped to the appropriate size. Both linear and nonlinear image registrations have enhanced the classifier's accuracy by around 4-5 percent when compared to no image registration. The implementation of the model is divided into three sections. In the first stage, a convolutional neural network is used to learn the feature map from brain MRI image space into the tumor marker area. A region-based convolutional neural network for tumor localization is presented in the second phase, followed by a region proposal network (RPN) to get the precise tumor contour. The segmentation and classification method is further expanded to create the structure of the next deep CNN and machine learning classifiers in series to enhance the accuracy of segmentation and classification output. The experimental results validate that the proposed deep CNN and SVM-RBF classifier achieved an accuracy of 98.3% and a dice similarity coefficient (DSC) of 97.8% on the task of classifying brain tumors as gliomas, meningioma, or pituitary using brain dataset-1, while on Figshare dataset, it achieved an accuracy of 98.0% and a DSC of 97.1% on classifying brain tumors as gliomas, meningioma, or pituitary.

The article "A Hybrid Approach Based on Deep CNN and Machine Learning Classifiers for the Tumor Segmentation and Classification in Brain MRI" was retracted in 2023. Reasons: signs of a paper mill; compromised peer review; unreliable results or conclusions.

We plan to expand this research in the future by experimenting with larger datasets and other tumor kinds. As a result, the suggested framework may be implemented as a useful system for doctors to give acceptable medical treatment methods for brain tumor early detection. The proposed model, however, still has flaws, such as a long computation time. The next study topic will be how to improve the algorithm and reduce the running time. Our work with CNN to determine the specific location of the tumor is likely to grow in the future with 3D brain imaging.

## Figures and Tables

**Figure 1:** Architecture of our proposed framework.

**Figure 2:** Linear registration of brain MRI adopted in this work.

**Figure 3:** Proposed CNN layout.

**Figure 4:** Region proposal network.

**Figure 5:** Working flow of deep CNN and machine learning classifiers.

**Figure 6:** Segmentation and classification of brain tumor based on deep CNN and SVM-RBF classifier.

**Figure 7:** AUC ROC curves for different tumor classes in brain dataset-1.

**Figure 8:** AUC ROC curves for different tumor classes in Figshare dataset.

**Figure 9:** Segmentation performance of the proposed deep CNN and machine learning classifiers in terms of MSE, PSNR, and BDE.

**Figure 10:** Segmentation performance of the proposed deep CNN and machine learning classifiers in terms of VOI, PRI, and GCE.

**Figure 11:** Performance of the proposed deep CNN SVM-RBF: (a) accuracy; (b) loss.

**Table 1:** Training and testing details of brain dataset-1.

Dataset		Total	Training	Testing
Brain dataset-1	Glioma	926	695	231
	Meningioma	937	702	235
	Pituitary	901	675	225
	Total	2764	2072	692

**Table 2:** Training and testing details of Figshare dataset.

Dataset		Total	Training	Testing
Figshare	Glioma	1426	1070	356
	Meningioma	708	531	177
	Pituitary	930	698	232
	Total	3064	2294	766

**Table 3:** Hyperparameter values used in our proposed model.

Hyperparameter	Value
Learning rate	0.00001
Number of epochs	100
Batch size	32
Optimizer	Adam

**Table 4:** Performance of the proposed model and machine learning classifiers on brain dataset-1.

Metrics	Tumor type	TP	TN	FP	FN	Sensitivity	Specificity	PPV	NPV	Accuracy	DSC
Method											
Deep CNN + random forest	Glioma	220	453	08	11	0.952	0.982	0.964	0.976	97.2%	95.8%
	Meningioma	222	448	09	13	0.944	0.980	0.961	0.971	96.8%	95.2%
	Pituitary	217	459	07	09	0.960	0.984	0.968	0.960	97.6%	96.4%

Deep CNN + SVM-RBF	Glioma	227	456	05	04	0.982	0.989	0.978	0.991	98.6%	98.0%
	Meningioma	232	451	06	03	0.987	0.986	0.974	0.993	98.0%	98.1%
	Pituitary	222	459	07	04	0.982	0.984	0.969	0.992	98.4%	97.5%

Deep CNN + ELM	Glioma	223	455	06	08	0.965	0.986	0.973	0.982	98.2%	96.9%
	Meningioma	226	450	07	09	0.961	0.984	0.969	0.980	97.6%	96.5%
	Pituitary	219	462	05	07	0.969	0.989	0.977	0.985	98.3%	97.3%

The article "A Hybrid Approach Based on Deep CNN and Machine Learning Classifiers for the Tumor Segmentation and Classification in Brain MRI" was retracted in 2023. Reasons: signs of a paper mill; compromised peer review; unreliable results or conclusions.

**Table 5:** Performance of the proposed model and machine learning classifiers on Figshare.

Metrics	Tumor type	TP	TN	FP	FN	Sensitivity	Specificity	PPV	NPV	Accuracy	DSC
Method											
Deep CNN + random forest	Glioma	343	399	11	13	0.963	0.973	0.968	0.968	96.8%	96.6%
	Meningioma	169	580	09	08	0.954	0.984	0.949	0.986	97.8%	95.2%
	Pituitary	221	524	10	11	0.952	0.981	0.956	0.979	97.3%	95.4%

Deep CNN + SVM-RBF	Glioma	348	401	09	08	0.977	0.978	0.974	0.980	97.7%	97.6%
	Meningioma	171	581	08	06	0.966	0.986	0.955	0.989	98.1%	96.0%
	Pituitary	225	528	06	07	0.970	0.988	0.974	0.986	98.3%	97.1%

Deep CNN + ELM	Glioma	341	397	13	15	0.957	0.968	0.963	0.963	96.3%	96.0%
	Meningioma	166	579	10	11	0.937	0.983	0.943	0.981	97.2%	94.0%
	Pituitary	220	521	13	12	0.948	0.975	0.944	0.977	96.7%	94.6%

**Table 6:** Performance of the proposed deep CNN and machine learning classifiers on brain dataset-1 and Figshare dataset with and without image registration.

Dataset	Preprocessing	Model	Sensitivity	Specificity	PPV	NPV	Accuracy	DSC
Brain dataset-1	Without image registration	Deep CNN + random forest	0.932	0.961	0.934	0.943	94.5%	92.4%
		Deep CNN + SVM-RBF	0.960	0.958	0.942	0.963	95.6%	93.3%
		Deep CNN + ELM	0.944	0.955	0.951	0.967	95.1%	94.6%
	With image registration	Deep CNN + random forest	0.951	0.982	0.964	0.969	97.2%	95.8%
		Deep CNN + SVM-RBF	0.983	0.986	0.973	0.992	98.3%	97.8%
		Deep CNN + ELM	0.965	0.984	0.972	0.982	98.0%	97.0%

Figshare dataset	Without image registration	Deep CNN + random forest	0.938	0.964	0.939	0.963	92.4%	91.8%
		Deep CNN + SVM-RBF	0.959	0.973	0.951	0.971	94.5%	93.2%
		Deep CNN + ELM	0.928	0.959	0.938	0.960	91.2%	90.4%
	With image registration	Deep CNN + random forest	0.956	0.979	0.957	0.977	97.8%	95.7%
		Deep CNN + SVM-RBF	0.971	0.984	0.967	0.985	98.0%	97.1%
		Deep CNN + ELM	0.947	0.975	0.950	0.973	96.7%	94.8%

**Table 7:** Comparative analysis of proposed method and previous related works.

Authors	Dataset	Model	Accuracy
Francisco et al. [40]	3064 MR images	Multipath CNN	97.3%
Çinar and Yıldırım [41]	253 MR images	CNN	97.2%
Hemanth et al. [42]	220 MR images	CNN	94.5%
Huang et al. [43]	3064 MR images	CNN	95.49%
Saxena et al. [44]	253 MR images	CNN models with transfer learning approach	95%
Ge et al. [49]	BraTS 2017	Multistream 2D CNN	88.82%
Ayadi et al. [45]	3064 MR images	Capsule-net	94.74%
Ghassemi et al. [46]	3064 MR images	GAN + ConvNet	93.01%
Ozyurt et al. [47]	500 MR images	SR-FCM-CNN	95.62%
Sultan et al. [48]	233 MR images	Deep CNN	96.13%
Our proposed model	Brain dataset-1: 2764 MR images	Deep CNN + SVM-RBF	98.3%
	Figshare dataset: 3064 MR images		98.0%

The article "A Hybrid Approach Based on Deep CNN and Machine Learning Classifiers for the Tumor Segmentation and Classification in Brain MRI" was retracted in 2023. Reasons: signs of a paper mill; compromised peer review; unreliable results or conclusions.

## Data Availability

*The data that support the findings of this study are openly available in the* Brain Tumor Classification (MRI) Dataset (available online: https://www.kaggle.com/sartajbhuvaji/brain-tumor-classification-mri and *Figshare dataset* doi:10.6084/m9.figshare.1512427.v5).
